# MicroRNA-205-5p Targets HMGB1 to Suppress Inflammatory Responses during Lung Injury after Hip Fracture

**DOI:** 10.1155/2019/7304895

**Published:** 2019-11-28

**Authors:** Xiaojie Yu, Xiaobin Chen, Tiansheng Sun

**Affiliations:** ^1^Department of Orthopaedics, The Second School of Clinical Medicine, Southern Medical University, Guangzhou, Guangdong 510515, China; ^2^Chinese PLA General Hospital, Medical Center 7, Department of Orthopedic Surgery, Beijing 100700, China

## Abstract

Hip fracture is the most common type of injury in elderly people and is associated with a high incidence of complications and risk of mortality. In these patients, subsequent pulmonary infection can contribute to the development of an acute lung injury, a consequence of the systemic inflammatory response induced by hip fracture. Although the crucial role of microRNAs (miRNAs) in inflammatory responses has been established, the functions of miRNAs in the inflammatory responses associated with lung injury after hip fracture remain poorly understood. In this study, we explored the potential role of miR-205-5p in lung injury after hip fracture in an *in vivo* hip fracture model and *in vitro* cultures of human pulmonary alveolar epithelial cells (HPAEpiC). An analysis of clinical serum samples revealed increased levels of miR-205-5p and high mobility group box 1 (HMGB1) after hip fracture. A bioinformatics analysis and dual-luciferase reporter assay identified *HMGB1* as a potential target of miR-205-5p. The overexpression of miR-205-5p clearly reduced the expression of HMGB1 and inhibited NF-*κ*B signaling, apoptosis, and proinflammatory cytokine production while enabling continued cell proliferation. Our results demonstrate that the upregulation of miR-205-5p suppresses inflammatory responses and promotes cell viability and proliferation by selectively targeting HMGB1 in the context of lung injury after hip fracture. Therefore, miR-205-5p may be an alternative target of therapeutic strategies for lung injury after hip fracture.

## 1. Introduction

Hip fracture is a common type of bone fracture in the elderly and is associated with high rates of mortality and a high incidence of complications that mainly result from immune disorders (e.g., rapid inflammatory response) [1]. Lung infection is the most severe of these complications, and previous studies have demonstrated that a hip fracture may subsequently contribute to a potentially fatal lung infection [2, 3]. For instance, hip fracture can affect the release of mitochondrial DNA release and induce lung injury via the TLR9/NF-kappa B (NF-*κ*B) pathway [4]. Moreover, the trauma associated with surgery, which is the current standard treatment strategy for hip fracture, could induce posttraumatic systemic inflammation and subsequent remote organ damage. For example, lung infection is the most common postoperative complication and has been associated with high hospitalization and mortality rates [5–8]. Although improvements in surgical techniques and hospital care and advanced prevention strategies have led to reductions in the incidence of complications after hip fracture, the risk of infectious and inflammatory lung injury after hip fracture remains very high [9]. Therefore, a detailed exploration of the molecular mechanisms involved in the progression of lung injury after hip fracture and the identification of a critical mediator as a potential therapeutic target in such cases are highly important.

Recent research has identified potentially crucial roles of microRNAs (miRNAs) in multiple pathological conditions, including cancers, cardiovascular diseases, and neurodegenerative diseases [10]. miRNAs regulate gene expression by directly targeting the 3′-untranslated region (3′-UTR) and inhibiting protein translation. Therefore, miRNAs contribute to most physiological and pathological processes by targeting the major molecular regulators. Studies have revealed that miRNAs may also play regulatory roles in remote organ damage caused by infection and inflammation [11–13]. For example, miR-146a was shown to act as a repressor of the inflammatory response during lipopolysaccharide- (LPS-) induced acute lung injury by inhibiting the expression of interleukin-1 receptor-associated kinase 1 (IRAK1) and tumor necrosis factor (TNF) receptor-associated factor 6 (TRAF6) [11, 12]. Another study demonstrated that human miR-921 mediates lung injury by targeting interleukin-37 (IL-37) expression [13]. miR-205-5p has been identified as a regulatory factor in several pathological conditions, including colon cancer [14], breast cancer [15], sepsis [16], and liver cancer [17].

Despite the above findings, the roles of miRNAs in the development of lung injury after hip fracture have not been well investigated. Therefore, we sought to identify the key miRNA in this process, as well as its potential target, with the aim of providing new insights into the underlying mechanism and identifying therapeutic strategies to treat lung injury after hip fracture. In this study, we explored the potential contribution of miR-205-5p to the progression of lung injury after hip fracture using both *in vivo* and *in vitro* models. We also investigated the expression of miR-205-5p and its regulatory effect on the inflammatory mediator HMGB1. Our results may provide new insights to inform the development of advanced therapeutic treatment and prevention strategies for lung injury after hip fracture.

## 2. Materials and Methods

### 2.1. Patients and Samples Collection

The clinical characteristics of patients with hip fracture who were included in this study are shown in Table 1. Serum samples were collected from all patients. Bone biopsies were conducted in accordance with the Updated Banff 07 Classification. The human experimental protocol was approved by the ethics committee of joint surgery of Zhuzhou Central Hospital (Hunan, China). The study protocol adhered strictly to the Code of Ethics of the World Medical Association (i.e., Declaration of Helsinki). All patients and their families participated voluntarily in the study and provided signed informed consent.

### 2.2. Experimental Animals

The animal experimental protocol was approved by the Animal Ethics Review Committee of Nanfang Hospital, Southern Medical University. Twenty male Sprague-Dawley (SD) rats were housed with unlimited access to food and water. After an acclimation period of >1 week, all of the animals were randomly assigned to one of two groups: control and fracture groups. The hip fracture model was established as described previously [18–20]. Briefly, the SD rats in the fracture group were anesthetized with sodium pentobarbital (60 mg/kg, intraperitoneally (i.p.)) and laid on the base of a blunt guillotine ramming apparatus. After identifying and marking the proximal femur, hip fracture was induced by dropping a blunt guillotine (weight: 500 g) from a height of 15 cm.

X-ray imaging was performed on Days 0 and 28 after hip fracture, and blood was collected at 0 h, at 8 h, and on Days 1, 7, 14, and 28. Lung tissues were collected on Day 28 after hip fracture. Changes in the statuses of the model animals were monitored by experienced technicians to avoid potential side effects such as peritonitis. At the end of the experiment (Day 28), the rats were anesthetized using 3% sodium pentobarbital i.p. and sacrificed by bleeding through the abdominal aorta. A postmortem examination was conducted to identify signs of peritonitis before further study.

### 2.3. Histomorphology Analysis

A section of lung tissue was treated with a fixative solution (4% formaldehyde and 1% glutaraldehyde in PBS, pH 7.4) and embedded in paraffin. A Leica SM2010R microtome (Leica, Shanghai, China) was used to cut the embedded tissue into 5-micrometer-thick slices, which were subjected to ethanol gradient dehydration and hematoxylin and eosin (H&E) staining. Finally, the slices were observed under a light microscope (Eclipse E100, Nikon, Japan; 40x magnification).

### 2.4. Immunohistochemical Staining

For immunohistochemical staining, fixed sections of lung tissue were blocked and then incubated with a primary antibody specific for HMGB1 (1 : 4000 dilution; ab79823, Abcam, UK) in 10% rabbit serum overnight at 4°C. The sections were then treated with a secondary antibody conjugated to horseradish peroxidase (1 : 10000 dilution; ab7090, Abcam). After the colorimetric reaction was completed, the sections were observed under a light microscope (Eclipse E100, Nikon; 40x magnification).

### 2.5. TUNEL Assay

Apoptosis was confirmed and quantified in tissue sections using the TUNEL assay. Tissue sections were stained with fluorescein-conjugated TUNEL (Click-iT™ TUNEL Alexa Fluor™ 594 Imaging Assay, Thermo Fisher Scientific, USA) according to the manufacturer's instructions [21]. The number of TUNEL-positive cells was counted in 30 sections per slide.

### 2.6. Cell Culture

Human pulmonary alveolar epithelial cells (HPAEpiC; BNCC337714, BeNa Culture Collection, Beijing, China) were cultured in Dulbecco's modified Eagle's medium (DMEM, 10566024, Gibco, USA) supplemented with 10% (*v*/*v*) fetal bovine serum (FBS, 10099-141, Gibco), 100 U/mL penicillin, 100 mg/mL streptomycin, and 2 mM glutamine. The cells were cultured at 37°C in an atmosphere of 5% CO_2_ and were passaged once they reached 70–80% confluency. HPAEpiC cells in the HMGB1-treated group were exposed to 15 *μ*g/mL HMGB1 [22]. Cells were cultured in DMEM medium containing 1% FBS and subjected to the following biochemistry analysis.

### 2.7. Cell Proliferation Assay

Cell proliferation was determined using Cell Counting Kit 8 (CCK-8) and an ethynyl-2-deoxyuridine incorporation assay (EdU Apollo DNA *in vitro* kit, RIBOBIO, Guangzhou, China) according to the manufacturer's instructions. For the CCK-8 assay, the cells were cultured at a density of 5 × 10^4^ per well in a 96-well plate. After a 24 h incubation to enable adherence, the cells were treated with CCK-8 solution for 2 h at 37°C. Subsequently, the absorbance at 450 nm was measured in each well using a multiwell plate reader (Multiskan MK3, Thermo Fisher Scientific).

For the EdU assay, the cells were treated with 100 *μ*L of EdU (50 *μ*M) for 2 h at 37°C at the end of each time point, then fixed in 100 *μ*L of 4% polyformaldehyde for 30 min at room temperature, treated with 50 *μ*L of glycine (2 mg/mL) for 5 min, and washed with 100 *μ*L of phosphate-buffered saline (PBS). After permeabilization with 0.5% Triton X, the cells were incubated in 1× Apollo solution for 30 min, in 100 *μ*L of 1× Hoechst 33342 solution (Cat. No. C10327, RiboBio, Shanghai, China) for another 30 min at room temperature in the dark, and washed with 100 *μ*L of PBS.

### 2.8. Apoptosis Analysis by Flow Cytometry and Hoechst 33258 Staining

Apoptosis was measured by the double staining of cells with Annexin V and propidium iodide (PI). After treating the culture plates with trypsin-EDTA, the detached cells were washed twice with PBS and resuspended in binding buffer (10 mM HEPES pH7.4, 150 mM NaCl, 5 mM KCl, 1 mM MgCl_2_, and 1.8 mM CaCl_2_) containing FITC-Annexin V (1 g/mL) for 20 min. PI (10 g/mL) was then added to the cell suspension. The cells were analyzed via flow cytometry, using the 488 nm and 575 nm wavelength channels to detect FITC and PI, respectively.

After the cells were transfected, 50 mL of cell stationary fluid (PBS containing 4% paraformaldehyde) was added. After 30-minute incubation at room temperature, the fluid was discarded and the samples were rinsed twice in PBS for 3 min per rinse. Next, a Hoechst 33258 staining solution (C1011, Beyotime, Beijing, China; final concentration: 20 *μ*M) was added for coverage at room temperature for 5 min. The dye solution was then discarded, and the samples were rinsed twice with PBS. Fluorescence microscopy was conducted at a wavelength of 460 nm.

### 2.9. Cell Cycle Analysis via Flow Cytometry

Cells were collected, washed with cold PBS buffer, and fixed in 70% ethanol at −20°C overnight. Subsequently, the cells were labeled with a staining solution containing 10 *μ*g/mL RNase A and 50 *μ*g/mL PI at 37°C for 30 min in the dark and then carefully washed with cold PBS. The cell cycle distribution was analyzed via flow cytometry with Cell Quest software (BD Biosciences, USA).

### 2.10. Analysis of RNA Expression by Real-Time PCR

The total RNA was isolated from cells using TRIzol (Invitrogen, USA). First-strand cDNA was then synthesized via reverse transcription and used in real-time PCR reactions, which were performed on an ABI 7500 Real-Time PCR System (Applied Biosciences, USA). Each assay was performed in triplicate. The following primer sequences were used: HMGB1, 5′-GTGCAAACTTGTCGGGAG-3′ (forward) and 5′-CGATACTCAGAGCAGAAGAGG-3′ (reverse); miR-205-5p, 5′-TCCTTCATTCCACCGGAGTCTG-3′ (forward) and 5′-CTCAACTGGTGTCGTGGAGTCGGCAATTCAGTTGAGCAGACTC-3′ (reverse); GAPDH, 5′-TGTTCGTCATGGGTGTGAAC-3′ (forward) and 5′-ATGGCATGGACTGTGGTCAT-3′ (reverse); and U6, 5′-CTCGCTTCGGCAGCACA-3′ (forward) and 5′-AACGCTTCACGAATTTGCGT-3′ (reverse). The relative expression levels of miR-205-5p and HMGB1 were calculated using the a 2^−ΔΔCt^ method. GAPDH and U6 were set as the internal controls, respectively.

### 2.11. In Silico Prediction and Dual-Luciferase Reporter Assay

The putative targets of miR-205-5p were predicted using Target Scan Release 7.2. Reporter vectors under the control of the wild-type and mutant human HMGB1 3′UTR were constructed using the pmirGLO vector backbone. A dual-luciferase assay reporter kit was used to detect firefly luciferase and *Renilla* luciferase signals.

### 2.12. Immunofluorescent Staining

Prior to immunofluorescent staining, the cells were fixed with 4% paraformaldehyde for 10 min and blocked with 5% FBS containing 0.5% Triton X-100 for 5 min. Subsequently, the cells were incubated at 4°C overnight in a solution containing primary antibodies specific for HMGB1 (1 : 4000 dilution, ab79823, Abcam) and NF-*κ*B p65 (1 : 1000, ab16502, Abcam). Subsequently, the cells were stained with an Alexa Fluor 488-conjugated anti-rabbit antibody and Alexa Fluor-564-conjugated anti-rabbit antibody. The cells were mounted on slides with mounting buffer containing DAPI. Immunofluorescence was detected using a fluorescence microscope.

### 2.13. Transfection of miR-205-5p Mimics and Inhibitor

miR-205-5p mimics and inhibitory and scramble (mock) miRNA were synthesized by GenePharma (Suzhou, China). HPAEpiC cells that had reached 80% confluency were transfected with miRNA via Lipofectamine 3000 reagent (Invitrogen, USA) according to the manufacturer's instructions.

### 2.14. Small Interfering RNA (siRNA) and Transfection Assays

*HMGB1*-specific siRNA was synthesized chemically, along with scramble siRNA as a negative control (NC). The siRNAs were transfected into cells using Lipofectamine 2000 reagent (Invitrogen) according to the manufacturer's instructions.

### 2.15. Western Blot Analysis

The samples were lysed with a protein lysis buffer containing 1% proteinase inhibitor and homogenized with an ultrasound homogenizer. After centrifugation for 10 min at 1200 g and 4°C, the supernatant was discarded and the total protein concentration in each sample was detected using a bicinchoninic acid (BCA) kit (PIERCE). Equal concentrations of protein per sample were prepared in 20 *μ*L of loading buffer and separated via sodium dodecyl sulfate-polyacrylamide gel electrophoresis (SDS-PAGE) at a constant voltage of 80 V. The separated proteins were then transferred to a polyvinylidene fluoride (PVDF) membrane (IPVH00010, Millipore, USA) at a constant voltage of 100 V for 90 min and then blocked in a 5% skim milk solution for 2 h. Then the band was cut according to the size of target band and incubated with primary rabbit antibodies specific for RAGE (1 : 1000, ab228861, Abcam), HMGB1 (1 : 4000, ab79823, Abcam), p65 (1 : 1000, ab16502, Abcam), and p-IkB*α*/IKB*α* (1 : 1000, ab133462/ab32518, Abcam) in Tris-buffered saline containing Tween-20 (TBS-T) overnight at 4°C. Next, the membranes were washed in TBS-T three times (10 min each) and incubated with a secondary antibody-linked HRP (1 : 10 000, ab7090, Abcam, UK). After adding an electrochemiluminescent solution, the membrane was imaged using a fluorescence imaging technique.

### 2.16. Cytokine and Chemokine ELISA Analysis

The concentrations of proinflammatory cytokines and chemokines in cell culture supernatants were evaluated using enzyme-linked immunosorbent assays (ELISAs) at 48 h after transfection. The supernatants were collected by centrifugation at 13000 g and 4°C for 10 min, and the total protein concentrations were measured using a DC protein assay (Bio-Rad, Hercules, CA, USA). The concentrations of HMGB1, IL-6, and TNF-*α* were then quantified by ELISA.

### 2.17. Data Analysis

Statistical calculations were performed using Prism 7 (GraphPad Software, Inc., USA). Data are presented as means ± standard deviations. Student's *t-*test was used for intergroup comparisons. Continuous data from multiple groups were analyzed using a one-way ANOVA, followed by Tukey's post hoc test. A Pearson correlation analysis was used to assess correlations between the expression of miR-205-5p and that of HMGB1 in human serum samples. Differences with *P* values <0.05 were considered statistically significant.

## 3. Results

### 3.1. Determination of Hip Fractures in SD Rats

X-ray images of rats in the control and hip fracture groups on Days 0 and 28 confirmed the successful establishment of the hip fracture model (Figure 1(a)). H&E staining of lung tissue sections revealed the main histologic differences in the hip fracture group relative to control group, including neutrophil marginalization around the lobules and cellulose-like necrosis in the arteries. Immunohistochemistry analysis revealed a remarkable increase in the HMGB1 level in the hip fracture group relative to the control group (Figure 1(b)). A TUNEL apoptosis assay indicated an increase in apoptosis in the hip fracture group relative to the control group (Figure 1(c)).

To explore the inflammatory responses in the SD rat model of hip fracture, we examined the concentrations of IL-6 and HMGB1 in serum samples via ELISA. Notably, we observed significant increases in HMGB1 in the fracture group at 8 h (*P* < 0.001) and on Days 1 (*P* < 0.001), 7 (*P* < 0.001), 14 (*P* < 0.001), and 28 (*P* < 0.001) after model induction. Similarly, we observed significant increases in IL-6 in the fracture group at 8 h (*P* < 0.001) and on Days 1 (*P* < 0.001), 7 (*P* < 0.01), and 14 (*P* < 0.01) after hip fracture. The serum level of miR-205-5p also increased at 8 h (*P* < 0.001) and on Days 1 (*P* < 0.001), 7 (*P* < 0.001), and 14 (*P* < 0.05) after hip fracture (Figure 1(d)). A Western blot analysis of lung tissue confirmed the dramatic increase in the level of HMGB1, as well as increases in NF-*κ*B p65, p-IkB*α*/IKB*α*, and RAGE in the hip fracture group relative to the control group (Figure 1(e)).

### 3.2. HMGB1 as a Target of miR-205-5p

Next, we determined the serum levels of miR-205-5p in lung injury after hip fracture patients against control group using quantitative real-time PCR (qPCR). Notably, miR-205-5p was upregulated in the sera of patients with lung injury (*P* < 0.01) after hip fracture relative to the controls. We also observed a significantly higher serum level of HMGB1 in patients with lung injury after hip fracture (*P* < 0.001) relative to controls (Figure 1(f)) and determined a positive correlation between the levels of miR-205-5p and HMGB1 in human serum (*R* = 0.684, Figure 1(g)).

Next, we conducted an *in silico* prediction analysis (miRBase, TargetScan, PicTar, and MiRanda) to identify the potential sites of binding between *HMGB1* mRNA and miR-205-5p. We determined that the 3′UTR of *HMGB1* mRNA includes a miR-205-5p-binding site that is conserved in mammals (Figure 1(h)). We then evaluated the effect of miR-205-5p on *HMGB1* expression using a luciferase reporter assay. Notably, an increase in miR-205-5p led to a significant decrease in luciferase activity under the control of the wild-type *HMGB1* 3′UTR relative to negative control. However, no significant difference from the control was observed when the predicted miR-205-5p-binding site in *HMGB1* mRNA was mutated (Figure 1(i)).

### 3.3. Effect of a miR-205-5p Mimic or Inhibitor in HPAEpiC Cells

To determine the effect of miR-205-5p on lung injury, miR-205-5p mimics or inhibitors (or mock) were transfected into HPAEpiC cells. We then evaluated the expression of miR-205-5p using qPCR, using U6 RNA as an internal control. miR-205-5p mimics significantly enhanced the expression of miR-205-5p (*P* < 0.01), while the miR-205-5p inhibitor dramatically decreased the expression of endogenous miR-205-5p (*P* < 0.01) relative to the controls. Moreover, the miR-205-5p mimic reduced the expression of *HMGB1* (*P* < 0.05), whereas the miR-205-5p inhibitor dramatically increased the expression of *HMGB1* (*P* < 0.001) by more than twofold (Figure 2(a)).

The CCK8 and EdU proliferation assays demonstrated that the transfection of the miR-205-5p mimic maintained cell proliferation, in contrast with the transfection of the miR-205-5p inhibitor (Figures 2(b) and 2(e)). Western blotting revealed significantly lower levels of HMGB1, NF-*κ*B p65, p-IkB*α*, and RAGE in the miR-205-5p mimic group and significantly higher levels of all four proteins in the miR-205-5p inhibitor group, relative to the miR-205-5p mock group (Figure 2(c)). Immunofluorescence staining of HMGB1 and p65 yielded similar results (Figure 2(d)).

Our apoptosis analysis revealed a significantly higher apoptosis rate in the miR-205-5p inhibitor group (*P* < 0.001; Figures 2(f) and 2(g)). Notably, transfection of the miR-205-5p inhibitor also disrupted the cell cycle distribution, with an increased percentage of cells in the G0/G1 phase (*P* < 0.01) and a corresponding decrease in the percentage of cells in the S phase (*P* < 0.01; Figure 2(h)). Furthermore, ELISA analyses revealed significant increases in the concentrations of HMGB1 (*P* < 0.01), IL-6 (*P* < 0.01), and TNF-*α* (*P* < 0.05) in the supernatants of cells in the miR-205-5p inhibitor group relative to the other two groups (Figure 2(i)).

### 3.4. The Effect of HMGB1 Administration and HMGB1 siRNA Transfection in HPAEpiC Cells

We validated the ability of HMGB1 siRNA to downregulate the expression of *HMGB1* using qPCR and western blotting. This RNA interference strategy significantly reduced the level of HMGB1 (*P* < 0.01) in the treated cells relative to the negative control cells (Figure 3(a)). Cell proliferation and apoptosis analyses revealed that the administration of HMGB1 significantly inhibited cell proliferation (*P* < 0.05) and promoted cell apoptosis (*P* < 0.01). However, transfection with siHMGB1 had no significant effect on either proliferation or apoptosis (Figures 3(b) and 3(d)–3(i)). Treatment with HMGB1 led to remarkable increases in the levels of p65, p-IkB*α*/IKB*α*, and RAGE relative to the control group, whereas decreased levels of all three proteins were observed in cells transfected with siHMGB1 (Figure 3(c)). An ELISA analysis confirmed significant increases in the levels of HMGB1 (*P* < 0.01), IL-6 (*P* < 0.01), and TNF-*α* (*P* < 0.01) in the supernatants of cells treated with HMGB1 group relative to the control, whereas the siRNA-mediated knockdown of HMGB1 significantly suppressed the expression of HMGB1 as expected (*P* < 0.01), as well as of IL-6 (*P* < 0.01) and TNF-*α* (*P* < 0.01; Figure 3(j)).

### 3.5. Effects of a miR-205-5p Mimic and HMGB1 Administration in HPAEpiC Cells

HPAEpiC cells transfected with a miR-205-5p mimic were subsequently treated with HMGB1, which led to a decrease in cell proliferation (*P* < 0.01) and an increase in apoptosis (*P* < 0.05) as indicated by flow cytometry and Hoechst 33258 staining analyses (Figures 4(a)–4(c)). Western blotting revealed decreased levels of HMGB1, NF-*κ*B p65, p-IkB*α*/IKB*α*, and RAGE in the miR-205-5p mimic + HMGB1 group relative to the HMGB1 group (Figure 4(d)). An ELISA analysis indicated significantly lower levels of HMGB1 (*P* < 0.01), IL-6 (*P* < 0.01), and TNF-*α* (*P* < 0.05) in the supernatants of miR-205-5p mimic + HMGB1 cells relative to the HMGB1 cells (Figure 4(e)).

## 4. Discussion

Recently, investigators have increasingly expressed interest in miRNAs, which selectively inhibit the expression of critical molecular compounds and thus contribute to the regulation of fundamental biological and physiopathological processes [23]. miRNAs also play modulatory roles in various cancers (e.g., breast, colon, liver, and cervical cancer), cardiovascular diseases (e.g., cardiac hypertrophy, hypertension, stroke, and arrhythmias), and neurodegenerative diseases (e.g., Alzheimer's disease, Huntington's disease, and Parkinson's disease) [24]. These pathological conditions are at least partially mediated by several miRNAs, suggesting that these elements may be useful as biomarkers or therapeutic targets. However, studies of the roles of miRNAs in inflammatory responses have been overshadowed by reports of the regulatory roles of miRNAs in cancers. To address this research gap, we investigated the functional role of a specific miRNA in the progression of the inflammatory response during lung injury after hip fracture.

Previous work established the ability of miRNAs to function as delay switches in the negative feedback regulation of inflammatory responses. For instance, miR-21 retards the inhibition of programmed cell death 4 (PDCD4) by activating NF-*κ*B [25]. Other studies have identified miR-146a as a modulator of immune suppression and miR-155 as a promoter of inflammatory responses [26–29]. In our study, we focused on the effect of miR-205-5p in inflammatory responses during lung injury after hip fracture, using clinical patient samples and cell culture experiments, as well as an *in vivo* rat model. Notably, we observed the upregulation of miR-205-5p in serum samples from patients and determined that the overexpression of miR-205-5p *in vitro* protected HPAEpiC cells from NF-*κ*B-mediated inflammatory responses induced by targeting HMGB1.

HMGB1 is produced and secreted by immune cells, such as macrophages and monocytes, and functions as a cytokine mediator in inflammatory responses. This protein exhibits multiple functions that depend on its subcellular location and may play a critical role in various pathological conditions [30, 31]. HMGB1 binds to Toll-like receptors (TLRs) and the receptor for advanced glycation end-products (RAGE) and thus activates NF-*κ*B signaling, which induces a variety of inflammatory responses. HMGB1 has been implicated to the progression of cancer, and one study described the ability of miR-200a to regulate liver cancer progression by targeting HMGB1 [32]. Moreover, Yao et al. demonstrated that miR-325 regulates HMGB1 in lung cancer [33].

In addition to the roles of other miRNAs, studies have demonstrated the involvement of miR-205-5p in the regulation of various proteins under different pathophysiological conditions [34–37]. In this study, we determined that the onset of inflammation due to hip fracture led to an increased level of HMGB1 and the upregulation of miR-205-5p. We subsequently identified HMGB1 as a direct target of miR-205-5p and observed that the overexpression of this miRNA reduced the levels of the NF-*κ*B signaling indicator p65, p-IkB*α*, RAGE, and the cytokines IL-6 and TNF-*α* in HPAEpiC cells, whereas the inhibition of miR-205-5p yielded the opposite effects. These results suggest that the miR-205-5p-mediated inhibition of HMGB1 led to the attenuation of NF-*κ*B signaling and subsequent inflammatory responses in HPAEpiC cells. We further observed that miR-205-5p affected apoptosis and cell proliferation in HPAEpiC cells. However, as these processes were not affected by siHMGB1, we cannot rule out the potential involvement of other pathways in this regulation. We plan to elucidate the exact mechanism in a future study. We note that treatment with HMGB1 enhanced NF-*κ*B signaling-induced inflammatory responses and apoptosis in HPAEpiC cells, thus supporting a direct relationship between miR-205-5p and HMGB1 in the suppression of inflammatory responses during lung injury after hip fracture. Our western blotting analysis revealed that treatment with miR-205 mimics remarkably reduced the level of HMGB1 in the cells. However, an ELISA analysis of protein levels in cell culture supernatants revealed no significant difference in the HMGB1 concentrations of the control and mimic-treated cultures. These findings further emphasize that the clinical effects of miR-205-5p and potential underlying mechanism will require further evaluation. Potentially, the application of a miR-205 mimic, miR-205 inhibitor, and siHMGB1 to a model of lung injury *in vivo* will elucidate this mechanism.

In conclusion, we have demonstrated that miR-205-5p attenuates the inflammatory responses and apoptosis induced by NF-*κ*B signaling and maintains the cell proliferative ability in the context of lung injury after hip fracture. The identification of HMGB1 as a specific target of miR-205-5 in this context provides a new direction for the development of small RNA-based therapies for lung injury after hip fracture.

## Figures and Tables

**Figure 1:** Determination of successful hip fracture in a Sprague-Dawley (SD) rat and of HMGB1 as the target of miR-205-5p. (a) Representative X-ray image of a SD rat model of hip fracture and control (1 : 1). (b) Representative hematoxylin and eosin-stained lung tissue sections and representative tissue sections stained immunohistochemically to detect HMGB1 are shown in the top and bottom panels, respectively (magnification, 40×). (c) Representative fluorescent images of tissues subjected to the TUNEL assay. Green and blue areas represent apoptotic cells and cell nuclei, respectively (magnification, 40×). (d) The relative expression levels of miR-205-5p and HMGB1 and IL-6 mRNA in the hip fracture and control groups were determined using qPCR. ^*∗*^*P* < 0.05, ^*∗∗*^*P* < 0.01, and ^*∗∗∗*^*P* < 0.001 vs. the control. (e) Western blot analysis of the levels of HMGB1, p65, p-IkB*α*/IkB*α*, and RAGE. Equal protein loading was verified using GAPDH or Lamin A as an internal control. (f) Relative levels of miR-205-5p and HMGB1 in serum samples from human patients relative to controls. ^*∗∗*^*P* < 0.01; ^*∗∗∗*^*P* < 0.001. (g) Correlation analysis between the levels of miR-205-5p and HMGB1 in human serum samples. (h) Predicted conserved miR-205-5p binding sites in HMGB1 mRNA. (i) Luciferase activity analysis of cells transfected with constructs encoding wild-type or mutated HMGB1 in the presence of miR-205-5p or NC. WT-3′UTR (+) indicates wild-type HMGB 3′UTR. WT-3′UTR (-) indicates mutant-3′UTR HMGB1. Mimics indicates miR-205-5p mimics. ^*∗∗*^*P* < 0.01 vs. the control.

**Figure 2:** Effects of a transfected miR-205-5p mimic or inhibitor in HPAEpiC cells. (a) The relative expression levels of miR-205-5p and HMGB1 were determined by qPCR. ^*∗*^*P* < 0.05, ^*∗∗*^*P* < 0.01, ^##^*P* < 0.01 and vs. the other two groups. (b) CCK8 assay of cell proliferation. The results represent the means of three independent experiments. ^*∗∗*^*P* < 0.01 and ^#^*P* < 0.05 vs. the other two groups. (c) Western blot analysis of the levels of HMGB1, p65, p-IkB*α*/IkB*α*, and RAGE. Equal protein loading was verified using GAPDH or Lamin A as internal controls. (d) The levels of HMGB1 and p65 were determined via immunofluorescence analysis (magnification, LSM 120×). (e) Representative micrographs of EdU-labeled samples from three groups (magnification, 10×) and (f) corresponding fluorescence images of samples stained with Hoechst 33258 (magnification, 20×). (g) Flow cytometric detection of apoptotic cells in samples double-stained with Annexin V-FITC and PI. ^*∗∗∗*^*P* < 0.001 vs. the other groups. (h) Images of a cell cycle analysis as determined by PI staining and flow cytometry. ^*∗∗*^*P* < 0.01 vs. the other groups. (i) The concentrations of HMGB1, IL-6, and TNF-*α* in cell supernatants were determined by ELISA. ^*∗*^*P* < 0.05, ^*∗∗*^*P* < 0.01, and ^*∗∗∗*^*P* < 0.001 vs. the other groups.

**Figure 3:** Effects of HMGB1 administration and siRNA-mediated inhibition in HPAEpiC cells. (a) The relative expression levels of miR-205-5p and HMGB1 were determined by qPCR. The control and siRNA control (siRNA-NC) groups are indicated by black and green bars, respectively. (b) Results of a CCK8 proliferation assay. The results are presented as the means of three independent experiments. ^*∗∗*^*P* < 0.05 and ^##^*P* < 0.05 vs. the other groups. (c) Western blot analysis of the levels of HMGB1, p65, p-IkB*α*/IkB*α*, and RAGE. Equivalent protein loading was verified using GAPDH or Lamin A as internal controls. (d) Representative micrographs of EdU-labeled samples from four groups and (e) corresponding fluorescence images of samples stained with Hoechst 33258. (f, h) Apoptotic cells were detected by flow cytometry and double-staining with Annexin V-FITC and PI. ^*∗∗*^*P* < 0.01 vs. the other groups. (g, i) Images of a flow cytometry-based cell cycle analysis of PI-labeled cells. ^*∗∗*^*P* < 0.01 and ^##^*P* < 0.01 vs. the other groups. (j) ELISA analysis of the levels of HMGB1, IL-6, and TNF-*α* in culture supernatants. ^*∗*^*P* < 0.05, ^*∗∗*^*P* < 0.01, and ^##^*P* < 0.01 vs. the other groups.

**Figure 4:** Effects of a transfected miR-205-5p mimic and HMGB1 treatment in HPAEpiC cells. (a) Fluorescence images of cells labeled with Hoechst 33258. (b) Apoptotic cells were detected by flow cytometry after double-staining with Annexin V-FITC and PI. ^*∗*^*P* < 0.05 vs. the other groups. (c) Images of a flow cytometric cell cycle analysis of PI-labeled cells.^*∗∗*^*P* < 0.01 and ^#^*P* < 0.05 vs. the other groups. (d) Western blot analysis of the levels of HMGB1, p65, p-IkB*α*/IkB*α*, and RAGE in cultured cells. (e) ELISA analysis of the concentrations of HMGB1, IL-6, and TNF-*α* in the culture supernatants. ^*∗*^*P* < 0.05 and ^*∗∗*^*P* < 0.01 vs. the other groups.

**Table 1:** Clinicopathological characteristics of patients included in the study sample.

	Hip fracture	Control
Variable	20	5
Sex		
Male	10	1
Female	10	4
Age		
60–69 years	6	1
70–79 years	6	3
80–89 years	6	1
90–99 years	2	0
Type of hip fracture		
Left femoral intertrochanteric fracture	9	
Right femoral intertrochanteric fracture	11	
Comorbid conditions		
Type II diabetes	9	
Hypertension	9	
Stroke complications	7	
Chronic lung diseases	2	

## Data Availability

The raw data of this study were available at the corresponding author upon reasonable request.

## Abbreviations

CCK8: Cell counting kit 8
ELISA: Enzyme-linked immunosorbent assay
H&E: Hematoxylin and eosin
HMGB1: High mobility group box 1
HPAEpiC: Human pulmonary alveolar epithelial cells
PDCD4: Programmed cell death 4
PI: Propidium iodide
RAGE: Receptor for advanced glycation end-products
SD: Sprague Dawley
siRNA: Small interfering RNA
TLRs: Toll-like receptors.

## References

[1] von Friesendorff M., McGuigan F. E., Wizert A. (2016). Hip fracture, mortality risk, and cause of death over two decades. *Osteoporosis International*.

[2] Lin J. C., Liang W. M. (2017). Mortality, readmission, and reoperation after hip fracture in nonagenarians. *BMC Musculoskeletal Disorders*.

[3] Zhang J. Z., Wang J., Qu W. C. (2017). Plasma mitochondrial DNA levels were independently associated with lung injury in elderly hip fracture patients. *Injury*.

[4] Gan L., Chen X., Sun T. (2015). Significance of serum mtDNA concentration in lung injury induced by hip fracture. *Shock*.

[5] Panula J., Pihlajamaki H., Mattila V. M. (2011). Mortality and cause of death in hip fracture patients aged 65 or older: a population-based study. *BMC Musculoskeletal Disorders*.

[6] Roche J. J., Wenn R. T., Sahota O., Moran C. G. (2005). Effect of comorbidities and postoperative complications on mortality after hip fracture in elderly people: prospective observational cohort study. *BMJ*.

[7] Lo I. L., Siu C. W., Tse H. F., Lau T. W., Leung F., Wong M. (2010). Pre-operative pulmonary assessment for patients with hip fracture. *Osteoporosis International*.

[8] Hao Z., Tiansheng S., Zhi L., Jianzheng Z., Xiaowei W., Jia L. (2014). Hip fracture aggravates systemic inflammation and lung injury in aged chronic cigarette smoke exposed rats. *Journal of Orthopaedic Research*.

[9] Haleem S., Lutchman L., Mayahi R., Grice J. E., Parker M. J. (2008). Mortality following hip fracture: trends and geographical variations over the last 40 years. *Injury*.

[10] Lekka E., Hall J. (2018). Non-coding RNAs in disease. *FEBS Letters*.

[11] Dai L., Zhang G., Cheng Z. (2018). Knockdown of LncRNA MALAT1 contributes to the suppression of inflammatory responses by up-regulating miR-146a in LPS-induced acute lung injury. *Connective Tissue Research*.

[12] Zeng Z., Gong H., Li Y. (2013). Upregulation of miR-146a contributes to the suppression of inflammatory responses in LPS-induced acute lung injury. *Experimental Lung Research*.

[13] Xu X. R., Liu C. Q., Feng B. S., Liu Z. J. (2014). Dysregulation of mucosal immune response in pathogenesis of inflammatory bowel disease. *World Journal of Gastroenterology*.

[14] Gulei D., Magdo L., Jurj A. (2018). The silent healer: miR-205-5p up-regulation inhibits epithelial to mesenchymal transition in colon cancer cells by indirectly up-regulating E-cadherin expression. *Cell Death and Disease*.

[15] Xiao Y., Li Y., Tao H. (2018). Integrin alpha5 down-regulation by miR-205 suppresses triple negative breast cancer stemness and metastasis by inhibiting the Src/Vav2/Rac1 pathway. *Cancer Letters*.

[16] Zhou W., Wang J., Li Z., Li J., Sang M. (2016). MicroRNA-2055b inhibits HMGB1 expression in LPS-induced sepsis. *International Journal of Molecular Medicine*.

[17] Lu J., Lin Y., Li F. (2018). MiR-205 suppresses tumor growth, invasion, and epithelial-mesenchymal transition by targeting SEMA4C in hepatocellular carcinoma. *The FASEB Journal*.

[18] Zhang H., Sun T., Liu Z., Zhang J., Wang X., Liu J. (2013). Systemic inflammatory responses and lung injury following hip fracture surgery increases susceptibility to infection in aged rats. *Mediators of Inflammation*.

[19] Qiu Y., Yang H., Lei B. (2014). Effects of three commonly used anesthetics on intraocular pressure in mouse. *Current Eye Research*.

[20] Bertera F. M., Di Verniero C. A., Mayer M. A., Bramuglia G. F., Taira C. A., Hocht C. (2009). Is urethane-chloralose anaesthesia appropriate for pharmacokinetic-pharmacodynamic assessment? Studies with carvedilol. *Journal of Pharmacological and Toxicological Methods*.

[21] Huo L., Fan Y., Wang H. (2019). Leukemia inhibitory factor receptor is involved in apoptosis in rat astrocytes exposed to oxygen-glucose deprivation. *BioMed Research International*.

[22] Wolfson R. K., Chiang E. T., Garcia J. G. (2011). HMGB1 induces human lung endothelial cell cytoskeletal rearrangement and barrier disruption. *Microvascular Research*.

[23] Di Leva G., Garofalo M., Croce C. M. (2014). MicroRNAs in cancer. *Annual Review of Pathology: Mechanisms of Disease*.

[24] Li Z., Rana T. M. (2014). Therapeutic targeting of microRNAs: current status and future challenges. *Nature Reviews Drug Discovery*.

[25] Sheedy F. J., Palsson-McDermott E., Hennessy E. J. (2014). Negative regulation of TLR4 via targeting of the proinflammatory tumor suppressor PDCD4 by the microRNA miR-21. *Nature Immunology*.

[26] Huffaker T. B., Hu R., Runtsch M. C. (2012). Epistasis between microRNAs 155 and 146a during T cell-mediated antitumor immunity. *Cell Reports*.

[27] Boldin M. P., Taganov K. D., Rao D. S. (2011). miR-146a is a significant brake on autoimmunity, myeloproliferation, and cancer in mice. *The Journal of Experimental Medicine*.

[28] Turner M. L., Schnorfeil F. M., Brocker T. (2011). MicroRNAs regulate dendritic cell differentiation and function. *The Journal of Immunology*.

[29] O’Connell R. M., Taganov K. D., Boldin M. P., Cheng G., Baltimore D. (2007). MicroRNA-155 is induced during the macrophage inflammatory response. *Proceedings of the National Academy of Sciences*.

[30] Yang R., Zhu S., Pischke S. E., Haugaa H., Zou X., Tonnessen T. I. (2018). Bile and circulating HMGB1 contributes to systemic inflammation in obstructive jaundice. *Journal of Surgical Research*.

[31] Kumari T., Kumar B. (2018). High-mobility group box 1 protein (HMGB1) gene polymorphisms and cancer susceptibility: a comprehensive meta-analysis. *Clinica Chimica Acta*.

[32] Li S., Huang Y., Huang Y. (2017). The long non-coding RNA TP73-AS1 modulates HCC cell proliferation through miR-200a-dependent HMGB1/RAGE regulation. *Journal of Experimental and Clinical Cancer Research*.

[33] Yao S., Zhao T., Jin H. (2015). Expression of MicroRNA-325-3p and its potential functions by targeting HMGB1 in non-small cell lung cancer. *Biomedicine and Pharmacotherapy*.

[34] Zhang P., Wang L., Rodriguez-Aguayo C. (2014). miR-205 acts as a tumour radiosensitizer by targeting ZEB1 and Ubc13. *Nature Communications*.

[35] Lin D., Halilovic A., Yue P. (2013). Inhibition of miR-205 impairs the wound-healing process in human corneal epithelial cells by targeting KIR4.1 (KCNJ10). *Investigative Opthalmology and Visual Science*.

[36] Orang A. V., Safaralizadeh R., Hosseinpour Feizi M. A., Somi M. H. (2014). Diagnostic and prognostic value of miR-205 in colorectal cancer. *Asian Pacific Journal of Cancer Prevention*.

[37] Qiao W., Chen L., Zhang M. (2014). MicroRNA-205 regulates the calcification and osteoblastic differentiation of vascular smooth muscle cells. *Cellular Physiology and Biochemistry*.

